The article "Exploring the Effects of Natural Capital Depletion and Natural Disasters on Happiness and Human Wellbeing: A Study in China" was retracted in 2025. Reasons: unreliable results or conclusions; a conflict of interest; concerns about the peer review; concerns about the citations.

# Exploring the Effects of Natural Capital Depletion and Natural Disasters on Happiness and Human Wellbeing: A Study in China

**DOI:** 10.3389/fpsyg.2022.870623

**Published:** 2022-05-23

**Authors:** Fami Lu, Muhammad Tayyab Sohail

**Affiliations:** ^1^School of Law and Humanities, China University of Mining and Technology, Beijing, China; ^2^School of Public Administration, Xiangtan University, Xiangtan, China

**Keywords:** organization, natural disasters, natural capital, happiness, human wellbeing

## Abstract

Since recent climate change has caused more natural disasters (NDs) than ever before, there is a worldwide concern that this could have both short-term and long-term economic and health consequences. This is perhaps the first attempt to explore the effects of natural capital (NC) and NDs on the human health and wellbeing of China over the period 1993–2020. The study has compiled data from World Bank, World Value Survey, UNDP, EM-DAT, and IMF for analysis. The empirical analysis is done by using the autoregressive distributed lag model. Empirical results prove that NC has a positive and significant effect on happiness, health, and human wellbeing in the long run. The results also show that NDs significantly reduce happiness and human wellbeing in the long run. The results recommend some important policy implications.

## Introduction

The depletion of natural capital (NC) all around the globe has irked policymakers, environmentalists, health experts, and empirics due to the mismanagement of natural resources and their adverse impact on health, the environment, and sustainable economic growth Arrow et al. (2012). To achieve sustainable development, natural resources must be used with great care so that these resources can be preserved for upcoming generations (Sohail et al., 2020; Liu et al., 2022). Goal No. 3, “good health and well-being,” of the sustainable development agenda 2030 of the United Nations (UN) posits that “Ensuring healthy lives and promoting well-being for all at all ages is crucial to sustainable development.” Even though the empirics have focused on the link between NC depletion and sustainable development; however, despite the importance of good health and wellbeing in achieving sustainable development, the literature is still in its infancy when it comes to the determinants of health and wellbeing. In this analysis, we try to plug this gap in the literature by examining the role of NC depletion and natural disasters (NDs) in affecting human health and wellbeing.

Happiness and human wellbeing studies have largely contributed to the literature of social sciences and economics. These studies gained significant attention due to increasing discontent among environmentalists, policymakers, and development economists. It is argued that economic development alone is not successful in providing the promised goals. The empirical research on happiness started with the work done by Easterlin (1974) and Hirsch (1976). In these studies, income has been used as a vital determinant of happiness. Afterward, it was recognized that income exerts little influence on happiness and quality of life. It is argued that income alone cannot enhance human wellbeing and happiness (Steptoe, 2019). Thus, it led to the exploration of other determinants that can contribute to ensuring happiness and wellbeing such as socioeconomic conditions, health, and quality of the environment. It is claimed that these determinants can influence happiness and wellbeing. Most specifically, connectedness with nature is also considered an important determinant of social and physiological wellbeing, health, and happiness (Zhang and Chen, 2019). The prevailing stock of literature revealed that spending time in nature enhances happiness and wellbeing (Kollamparambil, 2020). Kellert and Wilson (1983) argued that environmental quality significantly affects human psychology thus it is inherently associated with human wellbeing and happiness.

People living near beautiful scenery and green views are happier than those people living in a grimy and low-quality environment. The residents living near green environments experience higher wellbeing and life expectancy. In the case of Pennsylvania, Ulrich (1984) reported that the recovery rate of patients living in rooms with trees in the surrounding is higher than those patients living in rooms containing brick walls. Patients living near greenery required fewer medicines as they get healthier effects from the green environment. Similarly, the report published by California Energy Commission (2003) denoted that greenery and beautiful sight enhances the efficiency of workers and supports them to alleviate any undesirable health conditions. In the environment–happiness association, the important concern is environmental quality. Extreme moral hazards and climatic events occur as more dominant factors of happiness than money and income. These events can extremely damage psychological and physical health (Sekulova and Van den Bergh, 2016). Several studies have reported that environmental degradation is an alarming threat to human wellbeing, health, and happiness (Majeed and Ozturk, 2020).

As already mentioned, natural resources must be used cautiously to preserve them for future generations and to contribute to sustainable development. The adverse effects of natural resources extraction and the loss of welfare can only be minimized if these resources are reinvested in the development of other capital assets (Collier et al., 2010). It is worth mentioning here that the depleted NC must be used to develop humans and produce capital essential to promoting human health, wellbeing, and intergenerational welfare. However, the transformation of NC into human capital is yet to be established, although some empirical studies have observed that there is a negative association between natural resources, rents, and wealth growth (Koirala and Pradhan, 2020; van Krevel, 2021). As a result, natural resource extraction may lead to human capital development and speed up this development process (Lashitew and Werker, 2020), and consequently, promote human health and wellbeing.

A report from the WHO (2016) reveals that also 7 million deaths occur due to environmental pollution. According to the Disaster Risk Reduction Report (2004) of the United Nations, air pollution occurs due to a reduction in environmental quality that results from misuse of land, ambient contamination, and NDs. The rapid economic development and industrial revolution have deteriorated the environmental quality to an alarming magnitude; thus, culminating in key worldwide apprehensions. These apprehensions are related to rapid environmental variations, natural atmosphere disturbances, global warming, health risks, and the risk attached to overall human happiness and wellbeing (Ullah et al., 2020). The urban population increased sharply after 1950 leading to higher utilization of fertilizers and energy, thus creating a large number of gases such as nitrogen and carbon emissions. All these events transformed the world into a “new state” that becomes less appealing for human wellbeing and health. Thus, to preserve environmental amenity and human happiness, the environmental and NC-related issues have been incorporated into the research of human wellbeing, happiness, and health. The major share of greenhouse gases is composed of global warming and environmental pollution (Zafar et al., 2020). CO_2_ emissions are also considered a major cause of greenhouse gas emissions and NC depletion that constitute a major share of environmental deterioration. In view of IPCC (2014), the worldwide utilization of fossil fuels has significantly increased the energy demand, thus enhancing CO_2_ emissions. Anthropogenic events such as deforestation, burning of fossil fuels, and soil erosion are responsible for environmental degradation and NC depletion.

The United Nations adopted the agenda for SDGs in September 2015. The important goals of this agenda are sustainable growth of the ecosystem, sustainable development of cities, sustainability in consumption patterns, national equity, and reduction of poverty (Sohail et al., 2021a; Ullah et al., 2021). Engelbrecht (2009) reported that NC has a positive role in subjective wellbeing in high-income economies. Due to the incidence of NDs, the wellbeing and happiness of people and economic and social activities are likely to be disturbed. Literature reveals that tangible, intangible, direct, and indirect effects are expected from the NDs and the NC depletion. Akhter et al. (2020) reveal that losses from NC depletion and NDs are more powerful in the case of low-income economies.

Environment-related NDs are rapidly increasing with substantial influences on the animal, human, and NC. Most developing economies are facing the problems of NDs with growing concern that these events largely occur due to climatic variations (Van Aalst, 2006; Sohail et al., 2019a). Natural disasters lead to economic damage and result in large-scale mortalities. In 2009, 335 incidents of NDs were reported throughout the world with damages of 41 billion USD and almost 10,000 mortalities (Vos et al., 2010). In addition to the direct impacts on mortality, happiness, and health, NDs exert an indirect impact on human health and wellbeing through several mechanisms such as income constraints and lower access to health facilities during the phase of ND shocks. Particularly, exposure NDs during childhood could influence health trajectories by disturbing vital health-related investments. For instance, NDs may restrict children from getting immunizations timely. Furthermore, it may restrict the financial ability of households for investing in their children. An enormous body of literature highlights that childhood social-economic conditions and health experiences reveal long-term impacts on the mortality and health conditions of individuals (e.g., Leaning and Guha-Sapir, 2013; Rajapaksa et al., 2017; Dyregrov et al., 2018; Sohail et al., 2019b, 2021b). Exposure to several NDs including famines, tropical diseases, and epidemics significantly influences the wellbeing, happiness, and health outcomes of poor households (Sohail et al., 2014; Berlemann, 2016; Cui and Han, 2019; Maddison et al., 2020).

The above discussion highlights the significant contribution of NDs and NC in the determination of human wellbeing, happiness, and health conditions. In this perspective, this study aims to explore the influences of NC and NDs events on human wellbeing, happiness, and health. The study explores this nexus for China by using the autoregressive distributed lag (ARDL) approach for the period from 1993 to 2020. The findings of this study will help welfare economists, researchers, ecologists, development economists, and global organizations in designing policies. The study will help in formulating policies for improving health outcomes, happiness, and human wellbeing.

## Model and Methods

Natural disasters are a common occurrence in the world, and there is growing concern that they may become more frequent due to environmental issues. As a result, NDs have a significant impact on economic damage and can cause large-scale unhappiness and human death. Following standard literature by Freedy et al. (1993) and Datar et al. (2013), we assume that happiness, health, and human wellbeing have been determined by NC, NDs, CO_2_ emissions, financial development (FD), and technology. Time series models are used and are written as follows:


(1) $$\begin{array}{l} \begin{array}{ccc} Happiness_{t} & = & \lambda_{0}+\lambda_{1}NC_{t}+\lambda_{2}ND_{t}+\lambda_{3}CO_{2,t}+\lambda_{4}FD_{t} \end{array}\\ \begin{array}{c} \;+\lambda_{5}Technology_{t}+\varepsilon_{t} \end{array} \end{array}$$

(2) $$\begin{array}{l} \begin{array}{ccc} Health_{t} & = & \lambda_{0}+\lambda_{1}NC_{t}+\lambda_{2}ND_{t}+\lambda_{3}CO_{2,t}+\lambda_{4}FD_{t} \end{array}\\ \begin{array}{c} \;+\lambda_{5}Technology_{t}+\varepsilon_{t} \end{array} \end{array}$$

(3) $$\begin{array}{l} \begin{array}{ccc} HDI_{t} & = & \lambda_{0}+\lambda_{1}NC_{t}+\lambda_{2}ND_{t}+\lambda_{3}CO_{2,t}+\lambda_{4}FD_{t} \end{array}\\ \begin{array}{c} \;+\lambda_{5}Technology_{t}+\varepsilon_{t} \end{array} \end{array}$$

where the dependent variables Happiness, Health, and HDI represent national happiness, human health, and human development index, respectively; Happiness, Health, and HDI are the dependent variables that are determined by NC, NDs, CO_2_ emissions (CO_2_), FD, and technological innovation (Technology); λ_0_ is the intercept and ε_t_ is the error term. Natural capital is a stock of natural assets which increase happiness, human health, and wellbeing, thus λ_1_ will be positive. However, NDs have negative effects on national happiness, human health and wellbeing, thus an estimate of λ_2_ to be negative. The coefficient reported here is for long-run estimates. The next stage is to describe Equations (1)–(3) in an error–correction set-up so that we can also estimate the short-term effects. Therefore, the extended models are written as follows:


(4) $$\begin{array}{l} \Delta \text{Happines}{\text{s}}_{t}=\varphi_{0}+{\sum^{\text{​}}}_{k=1}^{n}\alpha_{1k}\Delta \text{Happines}{\text{s}}_{t-k}\\ +{\sum^{\text{​}}}_{k=0}^{n}\alpha_{2k}\Delta \text{N}{\text{C}}_{t-k}+{\sum^{\text{​}}}_{k=1}^{n}\alpha_{3k}\Delta \text{N}{\text{D}}_{t-k}\\ +{\sum^{\text{​}}}_{k=0}^{n}\alpha_{4k}\Delta \text{C}{\text{O}}_{2,t-k}+{\sum^{\text{​}}}_{k=1}^{n}\alpha_{5k}\Delta \text{F}{\text{D}}_{t-k}\\ +{\sum^{\text{​}}}_{k=0}^{n}\alpha_{6k}\Delta \text{Technolog}{\text{y}}_{t-k}+\lambda_{1}Happiness_{t-1}+\lambda_{2}NC_{t-1}\\ +\lambda_{3}ND_{t-1}+\lambda_{4}CO_{2,t-1}+\lambda_{5}FD_{t-1}+\lambda_{6}Technology_{t-1}\\ \begin{array}{c} +\lambda .ECM_{t-1}+\varepsilon_{t} \end{array} \end{array}$$

(5) $$\begin{array}{l} \Delta \text{Healt}{\text{h}}_{t}=\varphi_{0}+{\sum^{\text{​}}}_{k=1}^{n}\alpha_{1k}\Delta \text{Healt}{\text{h}}_{t-k}\\ +{\sum^{\text{​}}}_{k=0}^{n}\alpha_{2k}\Delta \text{N}{\text{C}}_{t-k}+{\sum^{\text{​}}}_{k=1}^{n}\alpha_{3k}\Delta \text{N}{\text{D}}_{t-k}\\ +{\sum^{\text{​}}}_{k=0}^{n}\alpha_{4k}\Delta \text{C}{\text{O}}_{2,t-k}+{\sum^{\text{​}}}_{k=1}^{n}\alpha_{5k}\Delta \text{F}{\text{D}}_{t-k}\\ +{\sum^{\text{​}}}_{k=0}^{n}\alpha_{6k}\Delta \text{Technolog}{\text{y}}_{t-k}+\lambda_{1}Health_{t-1}+\lambda_{2}NC_{t-1}\\ +\lambda_{3}ND_{t-1}+\lambda_{4}CO_{2,t-1}+\lambda_{5}FD_{t-1}+\lambda_{6}Technology_{t-1}\\ \begin{array}{c} +\lambda .ECM_{t-1}+\varepsilon_{t} \end{array} \end{array}$$

(6) $$\begin{array}{l} \Delta {\text{HDI}}_{t}=\varphi_{0}+{\sum^{\text{​}}}_{k=1}^{n}\alpha_{1k}\Delta {\text{HDI}}_{t-k}+{\sum^{\text{​}}}_{k=0}^{n}\alpha_{2k}\Delta {\text{NC}}_{t-k}\\ +{\sum^{\text{​}}}_{k=1}^{n}\alpha_{3k}\Delta {\text{ND}}_{t-k}+{\sum^{\text{​}}}_{k=0}^{n}\alpha_{4k}\Delta {\text{CO}}_{2,t-k}\\ +{\sum^{\text{​}}}_{k=1}^{n}\alpha_{5k}\Delta {\text{FD}}_{t-k}+{\sum^{\text{​}}}_{k=0}^{n}\alpha_{6k}\Delta {\text{Technology}}_{t-k}\\ +\lambda_{1}HDI_{t-1}+\lambda_{2}NC_{t-1}+\lambda_{3}ND_{t-1}\\ +\lambda_{4}CO_{2,t-1}+\lambda_{5}FD_{t-1}+\lambda_{6}Technology_{t-1}\\ \begin{array}{c} +\lambda .ECM_{t-1}+\varepsilon_{t} \end{array} \end{array}$$

In these three models, the coefficients assigned to first-differenced terms are short-term effects, but estimates of λ_1_ λ_6_ are the long-run effects. Specifications mentioned in Equations (4)–(6) are commonly referred to as the ARDL model (Pesaran et al., 2001). Following the study of Pesaran et al. (2001), who recommend two tests (*F*-test and ECM_t−1_) for the validity of long-run estimates. There are a few benefits of ARDL compared to other time–series estimators. The ARDL method is very simple and offers long and short-run effects in one step. The ARDL approach can be employed in a mixed order of integration. Moreover, the ARDL approach can be applied to small datasets, while Johansen's cointegration approach needs a large dataset for providing reliable estimation results. In the end, we also utilized some diagnostic tests, such as the Lagrange Multiplier (LM) test for serial correlation, Ramsey RESET test for model misspecification, Breusch–Pagan (BP) test for heteroskedasticity, and CUSUM and CUSUM-sq tests for stability of coefficient estimates.

### Data

The study uses time–series data for the period from 1993 to 2020 for exploring the effect of capital depletion and NDs on happiness, health, and wellbeing. Table 1 is composed of detailed information regarding definitions, symbols of variables, and sources of data. In this study, health is measured in terms of life expectancy at birth, and data is explored from the World Bank. Happiness is taken as a share of “people who are happy” and data is extracted from the World Value Survey. Wellbeing is measured by the human development index and the data is sourced from UNDP. Following Ouedraogo (2013), we use HDI as a measure of human wellbeing. Total natural resources rents as a percent of GDP are used to measure NDs and the data is taken from the World Bank. Natural disasters are measured as the “number of deaths” from disasters and data is explored from EM-DAT. Data for CO_2_ emissions and technology are explored from the World Bank while the data for the FD index is taken from the IMF. The detailed descriptive statistics are given in Table 2.

**Table 1:** Variables and definitions.

**Variables**	**Definitions**	**Sources**
Health	Life expectancy at birth, total (years)	World Bank
Happiness	Share of people who are happy	World Value Survey
HDI	Human development index	UNDP
NC	Total natural resources rents (% of GDP)	World Bank
ND	Number of deaths from disasters	EM-DAT
CO_2_	CO_2_ emissions (kt)	World Bank
FD	Financial development index	IMF
Technology	Patent applications, total	World Bank
	(residents and non-residents)	

**Table 2:** Descriptive statistics.

	**Health**	**Happiness**	**HDI**	**NC**	**ND**	**CO_**2**_**	**FD**	**Technology**
Mean	73.21	80.42	0.657	3.464	7.312	15.55	0.473	12.11
Median	73.27	79.94	0.661	2.983	7.160	15.67	0.467	12.25
Maximum	76.91	92.01	0.785	9.705	11.39	16.21	0.637	14.24
Minimum	69.49	67.00	0.531	1.047	5.869	14.78	0.321	9.836
SD	2.358	5.705	0.079	2.169	1.105	0.513	0.106	1.516
Skewness	−0.029	−0.055	−0.041	1.169	1.950	−0.167	0.228	−0.098
Kurtosis	1.748	3.099	1.684	3.876	7.973	1.374	1.646	1.668

## Results and Discussion

To confirm the presence of stationarity properties in data, the order of integration of variables has been checked. In this regard, Phillips Perron (PP) and Dickey–Fuller generalized least square (DF–GLS) tests have been used. Table 3 displays the outcomes of both unit root tests. The findings of both tests confirm the mixed order of integration among variables. According to of DF–GLS test, ND is stationary at a level while other variables are stationary at first difference. However, PP test gives us different results. It shows that health, happiness, ND, and NC are level stationary variables while human development index, CO_2_ emissions, FD, and technology are first difference stationary. Ullah et al. (2020) reported that in the presence of mixed order of integration, it is feasible to employ the ARDL approach. Table 4 is based on the short-run and long-run findings of ARDL models.

**Table 3:** Unit root testing.

	**PP**			**DF-GLS**		
	**I(0)**	**I(1)**	**Decision**	**I(0)**	**I(1)**	**Decision**
Health	−0.325	−2.641^*^	I(1)	−3.589^***^		I(0)
Happiness	−2.356	−3.655^**^	I(1)	−2.365^**^		I(0)
HDI	0.251	−4.325^***^	I(1)	0.365	−4.587^***^	I(1)
NC	−1.956	−6.355^***^	I(1)	−2.356^**^		I(0)
ND	−5.366^***^		I(0)	−5.325^***^		I(0)
CO_2_	−0.185	−2.756^*^	I(1)	−0.255	−2.566^**^	I(1)
FD	−0.254	−4.875^***^	I(1)	0.210	−4.325^***^	I(1)
Technology	−0.201	−4.336^***^	I(1)	−0.215	−3.754^***^	I(1)

*** *p < 0.01;*

** *p < 0.05; and*

* *p < 0*.

**Table 4:** ARDL estimates of health, happiness, and HDI.

	**Health**		**Happiness**		**HDI**	
**Variable**	**Coefficient**	***t*** **-Stat**	**Coefficient**	***t*** **-Stat**	**Coefficient**	***t*** **-Stat**
**Short-run**						
NC	0.011	0.469	0.092	0.476	0.007^*^	1.753
NC(−1)	0.013^***^	3.618	0.593^***^	3.079		
ND	−0.023^**^	2.051	−0.709^**^	2.410	−0.011	0.202
ND(−1)	0.013^**^	2.126			−0.002^*^	1.764
CO_2_	−0.079^**^	2.315	−2.291^***^	3.049	−0.035^*^	1.746
CO_2_(−1)	0.100^**^	2.241	1.602^***^	2.831	0.050^*^	1.910
FD	0.272^***^	4.440	1.509	0.110	0.134^**^	2.324
FD(−1)	−0.069	0.872	1.913	1.068	−0.117^*^	1.867
FD(−2)			1.966	1.169	0.104^*^	1.897
TECHNOLOGY	0.018	0.589	1.588^***^	3.556	0.003	0.495
TECHNOLOGY(−1)	−0.015	1.585	−0.480^***^	3.752		
**Long-run**						
NC	0.327^*^	1.804	0.920^***^	2.961	0.013^*^	1.828
ND	−0.130	0.622	−0.953^**^	2.407	−0.019^*^	1.752
CO_2_	−1.598^*^	1.713	−3.614^**^	2.465	−0.025	0.588
FD	2.466	0.673	3.509^***^	2.644	0.451^***^	3.011
TECHNOLOGY	2.638	0.911	0.145	0.056	0.012	1.025
C	7.116	0.787	6.107	1.421	4.013	0.026
**Diagnostics**						
F-test	7.144^***^^*^		8.352^***^		6.325^***^	
ECM(−1)	−0.587^**^	2.369	−0.644^***^	−9.252	−0.449^***^	−8.444
LM	0.689		0.698		1.858	
BP	0.635		1.287		0.258	
RESET	0.701		1.852		1.578	
CUSUM	S		S		S	
CUSUM-sq	S		S		S	

*** *p < 0.01;*

** *p < 0.05; and*

* *p < 0*.

In the long run, the findings of the health model reveal that NC and health are significantly and positively linked revealing that an increase in NC improves health quality. It shows that 1% intensification in NC improves health quality by 0.327% in the long run. However, NDs report a statistically insignificant effect on health quality in the long run. The CO_2_ emission is negatively attached to health quality displaying that 1% intensification in carbon emissions reduces health quality by 1.598% in the long run. Financial development and technology produce no significant influence on health quality in the long run.

The long-run findings of the happiness model report that NC is significantly and positively associated with happiness. It infers that 1% escalation in NC intensifies happiness by 0.920% in the long run. However, NDs report a significant and negative impact on happiness in the long term. It shows that a 1% increase in NDs reduces the level of happiness by 0.953% in the long run. Likewise, CO_2_ emissions also produce a significant and negative impact on happiness in the long run. It reveals that a 1% escalation in CO_2_ emissions reduces the level of happiness by 3.614% in the long run. In contrast, FD tends to significantly increase level of happiness in the long run. It reports that a 1% increase in FD increases the level of happiness by 3.509% in the long run. In the long run, the technology variable reports no significant impact on the level of happiness.

The long-run findings reveal that NC is significantly and positively associated with HDI. It reports that 1% rise in NC increases HDI by 0.013% in the long run. This finding is also supported by MacKerron and Mourato (2013), who noted that NC has a positive impact on health and human wellbeing. This means that nature might increase happiness by influencing human psychology. This finding is also supported by Apergis and Majeed (2021), who noted that people encircled by a green natural view are more likely to be happier than those living in a polluted environment. The findings of Kellert and Wilson (1983) noted that those populations that live in the natural environment have a manifest higher life expectancy. Our finding is also in line with Vemuri and Costanza (2006), who noted that NC is a key determinant of human wellbeing. As far as the relationship between NC depletion and human welfare is concerned, the lack of natural resources negatively impacts the wealth of the countries and leaves them with fewer resources to invest in health infrastructure, and decreases the overall health status of the society. A similar finding is also reported by Forson et al. (2017), Qureshi et al. (2019), and Koirala and Pradhan (2020).

However, NDs report a significant and negative impact on HDI in the long run. It infers that 1% intensification in NDs tends to reduce HDI by 0.019% in the long run. This finding is also backed by Prohaska and Peters (2019), who noted that NDs have a negative effect on health outcomes by increasing volumes of devastation and financial pressures. This means that NDs disturb the ecosystem, which in turn reduces human health, happiness, and wellbeing. This finding is also in line with Datar et al. (2013), who noted those NDs effects significantly on child health in India. It is widely recognized that environmental degradation may intensify the issue of NC depletion and ND trends (Bloom and Khanna, 2007). According to Sekulova and Van den Bergh (2016), instead of money and affluence, the happiness and wellbeing of the people are dominantly and negatively affected by natural calamities and natural depletion. Consequently, the ultimate impact of NDs can be seen on the physical and psychological wellbeing of the people. It is also well-documented that environmental degradation can prove fatal for human biological and psychological health, wellbeing, and happiness (Foudi et al., 2017; Sekulova et al., 2017).

The CO_2_ emissions and technology report an insignificant impact on HDI in the long run. This finding is also supported by Kampa and Castanas (2008), who noted that environmental pollution seriously damages human health. This means that a rapid increase in global warming has increased risks for human health, resulting in lowering happiness and human wellbeing. The emergence of technology innovation has improved the quality of life in China. However, FD tends to improve HDI in the long run. It infers that 1% rise in FD increases the level of HDI by 0.451% in the long run. The short-term findings reveal that NC reports a significant and positive impact on HDI only, while NDs report a significant and negative impact on health and happiness. Due to an increase in CO_2_ emissions, health, happiness, and HDI tend to decline in the short run. However, due to an increase in FD, health, happiness, and HDI tend to improve in the short run. Technology reports a significant and positive impact on happiness only in the short run. The findings of important diagnostic tests such as F-statistics, ECM, BP, LM, Ramsey RESET, CUSUM, and CUSUM-sq tests are given in the lower panel of Table 4. The long-run cointegration association is confirmed among variables in all three models as shown by the coefficient estimates of *F*-stat and ECM test. No issue of autocorrelation and heteroskedasticity is detected and all the models are correctly specified as shown by the statistically insignificant coefficient estimates of BP test, LM test, and Ramsey RESET test in all three models. The stability condition is also fulfilled in all three models as shown by the findings of CUSUM and CUSUM-sq tests.

## Conclusions

There is emergent concern that environmental changes lead to NC depletion and intensification of NDs such as floods, heavy rain, hurricane Mitch, and forest fires. It is fact that the worldwide deterioration in NC negatively influences the wellbeing and happiness of societies in the long run. This study contributes to the literature linking NC and NDs to health, wellbeing, and happiness. The objective of the study is to investigate the impact of NC and ND on human health, wellbeing, and happiness in China. The human development index is used to measure human wellbeing. However, life expectancy is used to measure health quality. Happiness is taken as the share of people who are happy. Besides these, the study has used carbon emissions, FD, and technology as control variables. Several findings have emerged from our results. First, NC has a significant positive impact on health, happiness, and wellbeing in the long run. Second, NDs report a significant and negative impact on happiness and wellbeing in the long run. Third, NC is positively associated with wellbeing only in the short run. Fourth, NDs report a significant and negative effect on health and happiness in the short run. In terms to control variables, we found that carbon emissions result in reducing happiness and health quality in the long run. While FD increases happiness and wellbeing in the long run. In contrast, technology reports a statistically insignificant impact on health, happiness, and wellbeing in the long run.

## Implications and Limitations

Findings suggest that governments should save natural resources on a priority basis. China's governments should establish policies to safeguard NC by changing consumer behavior to control the misuse of natural resources. As for natural resources, the government increased awareness and strict regulations to control illegal activities. Government should properly plan for the management of NC. The policymaker's recommendation for risk assessment and emergency awareness models that address the full impact of NDs on human health, happiness, and wellbeing. Policymakers should explore the efficiency of life and non-life insurance. Authorities should introduce smart technology to quantify and assess the effects on human health and the wellbeing of NDs. Mostly, pre- and post-disaster management policies are much needed for recurrent small-to-large level disasters.

This study has several limitations. Our study does not include child health, mental health, physical health, and economic performance; thus, these findings are traditional. Several new directions for future study arise from our study, including scrutinizing the role of NDs on child health, mental health, physical health, and economic performance. Additional research work on precise transmission mechanisms through which NDs influence economic effects and human health. Our study does not capture the world-specific policies and this study should also target global-level analysis.

## Data Availability Statement

The original contributions presented in the study are included in the article/supplementary material, further inquiries can be directed to the corresponding author/s.

## Author Contributions

FL and MT: conceptualization, investigation, supervision, writing, reviewing and editing, figure, formal analysis, and literature collection. Both authors contributed to the article and approved the submitted version.

## Conflict of Interest

The authors declare that the research was conducted in the absence of any commercial or financial relationships that could be construed as a potential conflict of interest.

## Publisher's Note

All claims expressed in this article are solely those of the authors and do not necessarily represent those of their affiliated organizations, or those of the publisher, the editors and the reviewers. Any product that may be evaluated in this article, or claim that may be made by its manufacturer, is not guaranteed or endorsed by the publisher.
